# An Efficient Ultrasound-Assisted Synthesis of Cu/Zn Hybrid MOF Nanostructures With High Microbial Strain Performance

This article has been retracted.

**DOI:** 10.3389/fbioe.2022.861580

**Published:** 2022-06-08

**Authors:** Gulnora Abdullaevna Abdieva, Indrajit Patra, Basim Al-Qargholi, Taher Shahryari, Narendra Pal Singh Chauhan, Mohammadreza Moghaddam-manesh

**Affiliations:** ^1^ Teaching Assistant, Department of Internal Medicine, Samarkand State Medical Institute, Samarkand, Uzbekistan; ^2^ An Independent Researcher, NIT, Durgapur, India; ^3^ Department of Biomedical Engineering, Al-Mustaqbal University College, Hilla, Iraq; ^4^ Department of Environmental Health Engineering, Faculty of Health, Social Determinants of Health Research Centre, Birjand University of Medical Sciences, Birjand, Iran; ^5^ Independent Researcher, Shrisela, India; ^6^ Petrochemistry and Polymer Research Group, Chemistry and Petrochemistry Research Center, Standard Research Institute, Tehran, Iran

**Keywords:** Cu/Zn MOF, hybrid nanostructures, ultrasound route, antibacterial nanostructures, antifungal activity

## Abstract

Metal organic frameworks (MOFs) are a promising choice for antibacterial and antifungal activity due to their composition, unique architecture, and larger surface area. Herein, the ultrasonic method was used to synthesize the Cu/Zn-MOF material as an effective hybrid nanostructure with ideal properties. SEM images were used to investigate the product’s morphology and particle size distribution. The XRD pattern revealed that the Cu/Zn hybrid MOF nanostructures had a smaller crystalline size distribution than pure Cu and Zn-MOF samples. Furthermore, the BET technique determined that the hybrid MOF nanostructures had a high specific surface area. TG analysis revealed that the hybrid MOF structures were more thermally stable than pure samples. The final product, with remarkable properties, was used as a new option in the field of antibacterial studies. Antibacterial activity was assessed using MIC and MBC against Gram negative and Gram positive strains, as well as antifungal activity using MIC and MFC. The antimicrobial properties of the synthesized Cu/Zn hybrid MOF nanostructures revealed that they were more effective than commercial drugs in some cases. This study’s protocol could be a new strategy for introducing new hybrid nanostructures with specific applications.

## 1 Introduction

Metal organic frameworks (MOFs) are a new class of nanostructured materials that have recently received special attention due to their properties (Ghanbari et al., 2020; He et al., 2022). These compounds have a wide range of potential applications, including electronic to biomedical applications (Al-Rowaili et al., 2018; Zhang et al., 2021; Zhu et al., 2022). Antibacterial applications are one of the applications of these compounds that distinguish nanostructures from other compounds (Kaur et al., 2021). The arrangement of the metal–organic framework, the nature of the metal, and the physicochemical properties of these compounds have all been significantly altered (Liu et al., 2021; Zhao et al., 2021).

According to research, the presence of beneficial physicochemical properties in MOF nanostructures such as high specific surface area, porosity, crystal structure, and pore distribution can influence antibacterial efficiency. As a result, introducing MOFs with such properties for antibacterial purposes is a significant challenge (Hasan et al., 2021).

MOF nanostructures can be combined with a wide range of compounds to form core-shell nanostructures, composites, and nanofibrous compounds. The physicochemical properties of the final compound are improved by this process. If the frameworks are integrated with each other to create hybrid structures, it appears that the properties of the final product will improve significantly (Sargazi et al., 2020; Liu and Tang, 2013; O'Neill et al., 2010).

It is also critical to select the right type of MOF nanostructure. Cu and Zn, as intermediate metals, have significant properties that influence product application due to their nature and active electron transfer. (Rodríguez et al., 2014; Restrepo et al., 20172017). These metals have been used as effective antibacterial candidates. Our findings revealed that there has been no previous report on the integration of Cu/Zn hybrid MOF nanostructures.

It is also critical to select a targeted route for the synthesis of MOF nanostructures. These compounds are synthesized in a variety of ways, including solvothermal, hydrothermal, and sol-gel (Guo et al., 2018; Sun et al., 2019). The results showed that sample synthesis in these methods requires a lot of energy and temperature, as well as a lot of time. The synthesis of MOF nanostructures using ultrasonic methods has recently received attention. This method is simple and efficient, and it can also affect the physicochemical properties of the final product (Abbasi et al., 2017; Zhang et al., 2022).

For the first time, Cu/Zn hybrid MOF nanostructures are synthesized using appropriate precursors *via* an efficient ultrasound route, and the final products are characterized by thermogravimetric analysis (TGA), X-ray diffraction (XRD), scanning electron microscopy (SEM), Fourier transform infrared spectroscopy (FTIR), CHNS/O elemental analyzer, and Brunauer–Emmett–Teller (BET) surface area analysis. The final products were found to be reasonably effective antimicrobial agents against pathogens such as Gram negative and Gram positive bacteria and fungi.

## 2 Experimental Section

### 2.1 Materials and Instrumentations

All materials were purchased commercially and used without further purification. Cu(NO_3_)_2_.6H_2_O was supplied by Sigma-Aldrich, and Zn(NO_3_)_2_.6H_2_O was obtained from Alfa Aesar (Shanghai, China). Sigma–Aldrich (St. Louis, MO, United States) provided the 2, 6-pyridine dicarboxylic acid. Adamas Reagent Co., Ltd. provided acetic acid (HAc, 99.5%) (Shanghai, China). The FT-IR spectra of samples were recorded in the transmission mode on a Nicolet AVATAR 360 FT-IR spectrophotometer with KBr powder as the sample matrix. For element analysis, X-ray diffraction (XRD) was performed using a Philips XPERT PRO Cu Ka radiation diffractometer. TGA was measured using a Netzsch Thermal analyzer STA 409 in an N_2_ atmosphere at a heating rate of 10°C/min. Surface morphologies of the prepared samples were identified using Hitachi S-4800 FE-SEM images on ITO-glass (Japan). The elemental CHN/O analyses were used to characterize the related elements. The BET surface areas of Cu/Zn hybrid MOF nanostructure samples were determined at 77 K using a Micromeritics TriStar II 3020 analyzer.

### 2.2 Synthesis of Cu-MOF Nanostructures

Solutions of Cu(NO_3_)_2_.5H_2_O (0.2 mmol; Mw: 232.6) and 2, 6-pyridine dicarboxylic acid (0.6 mmol; Mw: 167.1) were prepared in 35 ml of double-distilled water under ultrasound irradiation. The resulting solutions were placed in a Pyrex tube, and ultrasound irradiation was fixed at a frequency of 20 kHz for 20 min at a power of 190 W and a temperature of 30°C. Finally, after centrifugation, the prepared green crystals were washed thoroughly with DMF three times)and dried under an argon atmosphere.

### 2.3 Synthesis of Zn-MOF Nanostructures

The solutions including Zn(NO_3_)_2_.5H2O (0.2 mmol) and 2, 6- pyridine dicarboxylic acid (0.6 mmol) in 35 ml of double-distilled water were prepared under ultrasound irradiation. The resultant solution was then transferred to a Pyrex tube and subjected to the same conditions as in Section 2.2 (frequency: 20 kHz, reaction time: 20 min, and power: 190 W), at a temperature of 40 °C. Finally, the white crystals of Zn-MOF nanostructures were thoroughly washed three times with DMF and dried under an argon atmosphere.

### 2.4 Synthesis of Ni/Zn- Hybrid MOF Nanostructures

The Cu/Zn hybrid MOF nanostructures were developed using an ultrasound-assisted method. First, 0.03 g of Cu-MOF was dissolved in 20 ml of acetic acid (Sol. ***A***). Following that, in a separate tube, 0.03 g of Zn-MOF was dissolved in 35 ml of acetic acid (Sol. ***B***). Then, the Sol. ***B*** was added to the Sol. *A* at a temperature of 60°C under magnetic stirring at 230 rpm. The resultant solution was placed in an ultrasound bath under optimal conditions, including power of 240 W, time duration of 35 min, and temperature of 30°C. The crystals related to the formation of Ni/Zn hybrid MOF nanostructures were centrifuged and dried under an argon atmosphere.

### 2.5 Antimicrobial Activity

In antibacterial activity, Gram negative pathogenic strains including *Escherichia coli* (PTCC 1399) and *Salmonella enterica* subsp. *enterica* (PTCC 1709), Gram positive pathogenic strains including *Proteus mirabilis* (PTCC 1776) and *Rhodococcus equi* (PTCC 1633) and fungi including *Candida albicans* (PTCC 5027) that were prepared from the Persian Type Culture Collection (PTCC), Tehran, were used (Lu et al., 2021).

According to previous studies and CLSI (Clinical and Laboratory Standards Institute) guidelines M07-A9, M27-A2, and M26-A, broth micro dilution susceptibility and time-kill tests based on MIC (Minimum Inhibitory Concentration), MBC (minimum bactericidal concentration), and MFC (minimum fungicidal concentration) values were evaluated (Hosseinzadegan et al., 2020; Moghaddam-Manesh et al., 2020; Moghaddam-manesh et al., 2021).

## 3 Result and Discussion

### 3.1 Morphology and Size Distribution

The SEM images of Cu-MOF, Zn-MOF, and Cu/Zn hybrid MOF nanostructures are shown in Figure 1. According to the findings, there is strong evidence for aggregating particles in pure Cu- and Zn-MOF samples, and as a result, the particle morphologies are non-uniform. Nanostructures with a homogeneous morphology are synthesized in the Cu/Zn hybrid MOF nanostructure (Yang et al., 2017; Gao et al., 2019). As a result, the use of hybrid nanostructures has a significant impact on the final product’s morphology. The use of the best ultrasound method also had an impact on the morphology and size distribution of the samples synthesized in this study (Al-Attri et al., 2022). The samples synthesized in previous studies using conventional methods have a bulk size distribution, and the particles are dispersed as aggregates, which is important evidence (Bah et al., 2009; Zhang et al., 2018). In this study, the morphology and size distribution of the products were well affected by the synthesis of samples using the ultrasound route under optimal conditions, as well as the hybrid effects of nanostructures.

**FIGURE 1:** SEM image of the Cu-MOF **(A)**, Zn-MOF **(B),** and Cu/Zn hybrid MOF nanostructures **(C)**.

### 3.2 Thermal Stability

Thermal stability of Cu-MOF, Zn-MOF, and Cu/Zn hybrid MOF nanostructures is shown in Figure 2. According to the results, although the thermal patterns of all three samples have similar behavior, the stability of the Cu/Zn hybrid MOF nanostructures is higher than that of pure Cu and Zn nanostructures. It degraded in two stages: initially, from 65 to 350°C due to water loss and then from 350 to 500°C due to organic framework scission. It seems that the physicochemical effects of both Cu- and Zn-MOF nanostructures on the final hybrid structure are effective, which results in the creation of products with high thermal stability properties (Guo et al., 2017). The synthesis of samples with high stability properties significantly affects the application potential of the product (Chekol et al., 2018; Xia et al., 2019). The residual of the sample components disappears according to a regular pattern, which could be due to the loss of the linker, metal, and coordinated solvent.

**FIGURE 2:** Thermal behavior of the Cu-MOF **(A)**, Zn-MOF **(B),** and Cu/Zn hybrid MOF nanostructures **(C)**.

### 3.3 Crystallinity

X-ray diffraction patterns of Cu-MOF, Zn-MOF, and Cu/Zn hybrid MOF nanostructures are shown in Figure 3. Based on the results, the characteristic peaks of Cu-MOF and Zn-MOF are well observed in the final structure of Cu/Zn hybrid MOF nanostructures. According to the Debye–Scherrer equation, the average crystalline sizes of Cu-MOF and Zn-MOF are 70 and 65 nm, respectively. The wildness distribution of the diffraction patterns in the Cu/Zn-hybrid MOF nanostructures indicates the small size of the crystals. As an important result, the hybrid effects as well as the use of the optimal ultrasound conditions have led to the synthesis of samples with a small crystalline size distribution (Yang et al., 2019). Also, based on the results obtained from Xpert software, the crystallographic properties of the Cu/Zn hybrid MOF nanostructures are presented in Table 1.

**FIGURE 3:** XRD patterns of the Cu-MOF **(A)**, Zn-MOF **(B),** and Cu/Zn hybrid MOF nanostructures **(C)**.

**TABLE 1:** Crystallographic data for Cu/Zn hybrid MOF nanostructures.

Factor	Resulted data
Crystal structure	Hexagonal
Space group a (Å)	P4332
b (Å)	13.849
c (Å)	13.849
Alpha (°)	13.849
Beta (°)	90.000
Gamma (°)	90.000

### 3.4 Suggested Structures

FT-IR spectra of Cu-MOF, Zn-MOF, and Cu/Zn-MOF hybrid nanostructures are depicted in Figure 4. In all samples, a peak near 3,300 cm^−1^ confirmed the presence of coordinated water in the structure (Liu et al., 2008). The bands near 1,650–1700 cm^−1^ can be attributed to aromatic CH and COO groups, respectively (Mihaylov et al., 2015). The absorption bands around 900 cm^−1^ are attributed to the C-H bond, and the peaks in the range of 800–700 cm^−1^ may be assigned to Cu-O and Zn-O bonds. In Figure 4C, which indicates the FT-IR spectrum of Cu/Zn hybrid MOF nanostructures, all corresponding peaks related to pure Cu- and Zn-MOF hybrid nanostructures are observed, confirming the successful hybridization of Cu-MOF and Zn-MOF in the final structures (Zhong et al., 2017). CHNS/O elemental analysis of the Cu/Zn hybrid MOF nanostructures is shown in Figure 5, and the results from this Fig are presented in Table 2. As an important result, according to the FTIR data and CHNS/O analysis, the proposed structure of the Cu/Zn hybrid MOF nanostructures is shown in Figure 6.

**FIGURE 4:** FTIR spectra of the Cu-MOF **(A)**, Zn-MOF **(B),** and Cu/Zn hybrid MOF nanostructures **(C)**.

**FIGURE 5:** The CHNS/O elemental analysis for Cu/Zn hybrid MOF nanostructures.

**TABLE 2:** Elemental analysis of Cu/Zn hybrid MOF nanostructures using CHNS/O.

Element	Cu	Zn	C	H	N	O
Actual	—	—	42.45	1.89	6.78	31.04
Theoretical	8.80	9.05	42.42	1.92	6.79	31.02

**FIGURE 6:** Suggested structure for Cu/Zn-hybrid MOF nanostructures.

### 3.5 Adsorption/Desorption Behavior

Figure 7 shows the adsorption/desorption isotherms of Cu-MOF, Zn-MOF nanostructures, and Cu/Zn-hybrid MOF nanostructures synthesized by the ultrasound method. Based on classical adsorption/desorption isotherms, the behavior of pure Cu and Zn-MOF samples is similar to the second classical isotherm, which indicates a weak interaction between the nanostructure and the surface (Inagaki et al., 1996). Also, this type of isotherm showed that there is a slight porosity in the final products. On the other hand, the adsorption/desorption behaviors of hybrid nanostructures are similar to the first type of isotherms assigned to porous systems (Poyet, 2009; Yu et al., 2021). According to the BET results, the Cu/Zn hybrid MOF nanostructure sample has a specific surface area of about 1,400 m^2^/g, while the surface areas of Cu-and Zn-MOF nanostructures are 425 and 560 m^2^/g, respectively. As an important result, the hybrid nanostructures can be influenced by the adsorption/desorption behavior and specific surface area of the samples. The synthesis of nanostructures with the desired specific surface facilitates the conditions of these nanostructures for antibacterial applications.

**FIGURE 7:** N_2_ Adsorption/desorption of the Cu-MOF **(A)**, Zn-MOF **(B),** and Cu/Zn hybrid MOF nanostructures **(C)**.

### 3.6 Antimicrobial Activity

Table 3 shows the minimum inhibitory concentration, bactericidal concentration, and fungicidal concentration results due to the antibacterial and antifungal activity of Cu-MOF, Zn-MOF, and Cu/Zn hybrid MOF. The compounds had an effect on all Gram negative and Gram positive bacteria and fungal strains, according to the findings. The comparison of the results shows that the Cu/Zn hybrid MOF had a better effect by combining Cu-MOF and Zn-MOF in its structure. Because of their porous crystalline frameworks of bimetallic centers and organic linkers, as well as multiple covalent bonds, they are an important key player in inhibiting or killing microorganisms. Most microorganisms have negatively charged cell membranes that are easily attracted electrostatically by the metallic centers of MOFs, resulting in cytoplasmic membrane disruption and subsequent leakage of cytoplasmic constituents, which leads to cell death.

**TABLE 3:** Antibacterial activities against Gram negative strains and Gram positive strains and antifungal activities of Cu-MOF, Zn-MOF, and Cu/Zn hybrid MOF nanostructures.

Synthetic compound/drug			Bacteria				Fungi
			Gram negative strains		Gram positive strains		
			1,399	1709	1776	1,633	5,027
Cu-MOF		MIC	64	512	128	128	256
		MBC/MFC	128	1,024	256	256	256
Zn-MOF		MIC	128	1,024	256	128	256
		MBC/MFC	256	2048	512	256	512
Cu/Zn hybrid MOF		MIC	64	256	32	64	64
		MBC/MFC	64	512	64	128	128
Drug	A	MIC	—	8	16	8	32
		MBC/MFC	—	16	16	16	64
	B	MIC	8	4	1	2	—
		MBC/MFC	16	8	2	4	—

MIC, MBC, and MFC values reported as μg/mL; MBC for bacteria and MFC for fungi; drug for bacteria A: penicillin, B: gentamicin, for fungi: A: terbinafine, B: tolnaftate.

The antibacterial and antifungal activities of the compounds were compared with commercial drugs such as penicillin and gentamicin (as antibacterial drugs), terbinafine and tolnaftate (as antifungal drugs). Penicillin had no effect on *Escherichia coli*, but Cu-MOF, Zn-MOF, and Cu/Zn-hybrid MOF, particularly Cu/Zn-hybrid MOF with MBC: 64 μg/ml, had a strong effect. Tolnaftate had no effect on *Candida albicans*, but Cu-MOF, Zn-MOF, and Cu/Zn-hybrid MOF, particularly Cu/Zn-hybrid MOF with MFC: 128 gg/mL, had a significant effect.

## Conclusion

In this study, a novel Cu/Zn-MOF nanostructure with a narrow particle size distribution, high surface area, significant porosity, and high thermal stability was synthesized by the incorporation of pure Cu and Zn MOF nanostructures. The products were optimized under ultrasound irradiation and used as a novel candidate in antibacterial studies. In conclusion, the results of the antimicrobial and antifungal activities of the synthesized compounds showed that the compounds have acceptable antibacterial and antifungal properties, and the highest effect was related to Cu/Zn hybrid MOF, which has Cu-MOF and Zn-MOF in its structure.

## Data Availability

The raw data supporting the conclusion of this article will be made available by the authors without undue reservation.
